The article "Haplotype analysis on correlation between transcription factor 7-like 2 gene polymorphism and breast cancer risk" was retracted in 2024. Reasons: plagiarism; overlap with other authors' work; lack of ethics approval or compliance.

# Haplotype analysis on correlation between transcription factor 7-like 2 gene polymorphism and breast cancer risk

**DOI:** 10.1186/s12885-021-08571-4

**Published:** 2021-08-02

**Authors:** Yang Wang, Xiaojuan Men, Yongxue Gu, Huidong Wang, Zhicai Xu

**Affiliations:** Department of Galactophore Surgery, Weifang People’s Hospital, No.151 Guangwen Street, Kuiwen District, Weifang, 261041 Shandong Province People’s Republic of China

**Keywords:** Haplotype, Transcription factor 7-like 2, Polymorphisms, Breast cancer, Interaction

## Abstract

**Background:**

Up to now, limited researches focused on the association between transcription factor 7-like 2 gene (*TF7L2*) gene single nucleotide polymorphisms (SNPs) and breast cancer (BC) risk. The aim of this study was to evaluate the associations between *TF7L2* and BC risk in Chinese Han population.

**Methods:**

Logistic regression model was used to test the correlation between polymorphisms and BC risk. Strength of association was evaluated by odds ratio (OR) and 95% confidence interval (CI). Generalized multifactor dimensionality reduction (GMDR) was applied to analyze the SNP-SNP and gene-environment interaction.

**Results:**

Logistic regression analysis indicated that the BC risk was obviously higher in carriers of rs1225404 polymorphism C allele than that in TT genotype carriers (TC or CC versus TT), adjusted OR (95%CI) =1.40 (1.09–1.72). Additionally, we also discovered that people with rs7903146- T allele had an obviously higher risk of BC than people with CC allele (CT or TT versus CC), adjusted OR (95%CI) =1.44 (1.09–1.82). GMDR model was used to research the effect of interaction among 4 SNPs and environmental factors on BC risk. We discovered an important two-locus model (*p* = 0.0100) including rs1225404 and abdominal obesity, suggesting a potential gene–environment correlation between rs1225404 and abdominal obesity. In general, the cross-validation consistency of two-locus model was 10 of 10, and the testing accuracy was 0.632. Compared with subjects with normal waist circumference (WC) value and rs1225404 TT genotype, abdominal obese subjects with rs1225404 TC or CC genotype had the highest BC risk. After covariate adjustment, OR (95%CI) was 2.23 (1.62–2.89). Haplotype analysis indicated that haplotype containing rs1225404-T and rs7903146-C alleles were associated with higher BC risk.

**Conclusions:**

C allele of rs1225404 and T allele of rs7903146, interaction between rs1225404 and abdominal obesity, rs1225404-T and rs7903146-C haplotype were all related to increased BC risk.

## Introduction

Breast cancer (BC) is the main cause of death for women all over the world and is a major public health problem [1, 2]. Its rapidly increasing mortality is influencing women in developing countries, especially Chinese women [3, 4]. According to the data published by China Cancer Center in 2018, there were 278,900 newly diagnosed BC patients in China, and 66,000 BC patients died in 2014 [5]. The pathogeny of BC involved various factors including smoking, diet, estrogen exposure, menstrual disorder, BC family history, etc. [6, 7]. Approximately 5–10% of all BC cases are hereditary [8].

The transcription factor 7-like 2 (*TCF7L2*) gene is located at human chromosome 10q25.3, 215.9 kb long, with 17 identified extrons. Previous studies have showed the relationship between *TCF7L2* gene and common diseases such as type 2 diabetes mellitus (T2DM) [9], diabetic nephropathy (DN) [10], nonalcoholic fatty liver [11] and some cancers [12, 13]. The relationship between single nucleotide polymorphism (SNPs) of *TCF7L2* gene and BC risk was also reported in German [14], Hispanic [15], United States [16, 17] and Chinese population [18]. At present, there are few studies on the association between TCF7L2 SNPs and BC susceptibility. Additionally, BC development was the outcome of complicated interaction among gene and environment. Therefore, the purpose of this study is to evaluate the relationship between *TCF7L2* gene polymorphism and BC risk, as well as the effect of SNP-SNP and gene-environment interactions on BC risk in Chinese Han population.

## Materials and methods

### Study population

Subjects were recruited continuously from Weifang People’s Hospital from June 2012 to July 2018. A total of 1252 participants with an average age of 51.7 ± 11.7 years were selected, involving 622 BC patients and 630 controls. Patients who had be treated by chemotherapy or radiotherapy (to ensure the accuracy of our information collection) or had other cancers were removed. All patients had a histologic and clinical diagnosis of BC. The control group was matched by sex, age, and ethnic background, while controls with BC family history and any type of others cancer were excluded. All study protocols of the current study were approved by ethics committee of Weifang People’s Hospital.

### Genotyping methods

SNP selection rules as follows: we selected those SNPs which were not well studied previously, and minor allele frequency (MAF) of those selected SNPs were greater than 2%. We selected 4 SNPs of *TCF7L2* gene: rs1225404, rs12255372, rs7903146 and rs11196205. According to instructions of DNA Blood Mini Kit (Qiagen, Hilden, Germany), 3 ml EDTA-processed blood samples were extracted from all subjects for DNA extraction, and DNA was preserved at − 20 °C before use. PCR-based restriction fragment length polymorphism was used for the selected four SNPs genotype. Primers applied in our research are displayed in Table 1.

**Table 1:** Description and primer sequences used for genotyping for 4 SNPs within *TCF7L2* gene

SNP ID	Chromosome	Functional Consequence	Nucleotide substitution	Primer sequences
rs1225404	10:113154906	Intron variant	T > C	F: 5′- ACGTTGGATGTTCAGTGCTGCGGTTCTTAG-3′ R: 5′- ACGTTGGATGACACTCACACTCACGCCTTC-3′
rs12255372	10:113049143	Intron variant	G > T	F: 5′- CTTGAGGTGTACTGGAAACTAAGGC-3′ R: 5′- CTGTCTATTTGGCATTCAAATGGA-3′
rs7903146	10:112998590	Intron variant	C > T	F: 5′-CTGAACAATTAGAGAGCTAAGCACTTTTTAGGTA-3′ R: 5′- TTTCACTATGTATTGTTGCCAGTCAGCAAACAC-3′
rs11196205	10:113047288	Intron variant	G > T	F: 5′- GAAAGT TCTCAACATTTATAACTTCG-3′ R: 5′- TTTGCCCAATAATATGCCATGAAA-3′

### Statistical analysis

In this study, the means and standard deviation (SD) were calculated for continuous variables with normal distribution, and the percentage was calculated for categorical variables. The χ^2^ test was used for comparison for categorical variables and *t-* test was used for comparison of continuous variables. The Hardy-Weinberg equilibrium (HWE) and the relationship between *TCF7L2* gene SNPs and BC susceptibility were evaluated by SNPStats (https://www.snpstats.net/). The interaction among four SNPs and gene- abdominal obesity interaction was detected by generalized multifactor dimensionality reduction (GMDR). Logistic regression stratified analysis was used to test the interaction effect found in GMDR results. The consistency of cross validation, accuracy of test balance and sign test were calculated to evaluate the interaction of each selection. Haplotype analysis for SNPs was performed by SHEsis software (http://shesisplus.bio-x.cn/).

## Results

A total of 1252 subjects with an average age of 51.7 ± 11.7 years were selected, including 622 BC cases and 630 controls. The characteristics of subjects stratified by case and control are shown in Table 2. The fertility rate of more than 3 children in controls was significantly higher than that in cases, and there were also differences in average WC, menarche age and menopause age between two groups.

**Table 2:** General characteristics of 1252 study participants in case and control group

Variables	BC patients (*n* = 622)	Normal group (*n* = 630)	*p-*values
Age (year) (Mean ± SD)	52.2 ± 11.7	51.3 ± 12.1	0.181
Age at menarche (years) (Mean ± SD)	13.6 ± 3.7	14.2 ± 2.6	0.0009
Age at menopause (years) (Mean ± SD)	48.3 ± 9.6	49.4 ± 10.1	0.048
Menopausal status N (%)			0.532
Premenopausal	301 (48.4)	316 (50.2)	
Postmenopausal	321 (51.6)	314 (49.8)	
WC (cm) (Mean ± SD)	84.5 ± 16.2	82.2 ± 15.3	0.0099
BMI (kg/m^2^) (Mean ± SD)	24.1 ± 9.1	23.2 ± 9.5	0.087
Number of children (≥3) N (%)	167 (26.8)	199 (31.6)	0.065

All genotypes in control group were distributed according to HWE (*p* > 0.05). The allele frequency of rs1225404- C and rs7903146- T in BC group was significantly higher than that in control group (29.9% versus 20.0 and 28.8% versus 19.4%). Logistic regression analysis indicated that the BC risk was higher in carriers of rs1225404 polymorphism C allele than that of TT genotype carriers (TC+ CC versus TT), adjusted OR (95%CI) =1.40 (1.09–1.72). Additionally, we also found that participants with rs7903146- T allele had an obviously higher risk of BC than participants with rs7903146- CC genotype (CT+ TT versus CC), adjusted OR (95%CI) =1.44 (1.09–1.82) (Table 3).

**Table 3:** Genotype and allele frequencies of 4 SNPs between case and control group

SNP	Genotypes and Alleles	Frequencies N (%)		OR (95%CI) ^a^	*P*-values
		Control (*n* = 622)	Case (*n* = 630)		
rs12255372					
	GG	361 (58.0)	331 (52.5)	Ref	
	GT	224 (36.0)	247 (39.2)	1.21 (0.90–1.63)	
	TT	37 (6.0)	52 (8.2)	1.30 (0.83–1.87)	
	G	946 (76.0)	909 (72.1)	Ref	
	T	298 (24.0)	351 (27.9)	1.23 (0.87–1.68)	
HWE test for controls					0.774
rs1225404					
	TT	404 (65.0)	320 (50.8)	Ref	
	TC	187 (30.1)	243 (38.6)	1.33 (1.12–1.60)	
	CC	31 (5.0)	67 (10.6)	1.54 (1.07–2.07)	
	T	995 (80.0)	883 (70.1)	Ref	
	C	249 (20.0)	377 (29.9)	1.40 (1.09–1.72)	
HWE test for controls					0.128
rs11196205					
	GG	357 (57.4)	323 (51.3)	Ref	
	GT	220 (35.4)	245 (38.9)	1.14 (0.83–1.51)	
	TT	45 (7.2)	62 (9.8)	1.22 (0.71–1.77)	
	G	934 (75.1)	891 (70.7)	Ref	
	T	310 (24.9)	369 (29.3)	1.18 (0.78–1.60)	
HWE test for controls					0.172
rs7903146					
	CC	409 (65.8)	325 (51.6)	Ref	
	CT	184 (29.6)	247 (39.2)	1.41 (1.16–1.69)	
	TT	29 (4.7)	58 (9.2)	1.52 (1.06–2.01)	
	C	1002 (80.6)	897 (71.2)	Ref	
	T	242 (19.4)	363 (28.8)	1.44 (1.09–1.82)	
HWE test for controls					0.162

^a^Adjusted for gender, age, age at menarche, age at menopause, number of children and WC

GMDR model was used to evaluate the effect of SNP- SNP and gene- abdominal obesity interaction on BC risk. Table 4 shows the results obtained from GMDR analysis. We found an important two-locus model (*p* = 0.0100) including rs1225404 and abdominal obesity, suggesting a potential gene–environment correlation between rs1225404 and abdominal obesity. In general, the cross-validation consistency of two-locus model was 10 of 10, and the testing accuracy was 0.632. Logistic regression was used to analyze the interaction between rs1225404 and abdominal obesity to get the odds ratio and 95%CI of the combined effect of rs1225404 and abdominal obesity on BC risk. Compared with subjects with normal WC value and rs1225404 genotype TT, abdominal obese subjects with rs1225404 genotype TC or CC had the highest BC risk. After covariate adjustment, OR (95%CI) was 2.23 (1.62–2.89) (Fig. 1).

**Table 4:** GMDR analysis on the best SNP–SNP and gene- abdominal obesity interaction models

Locus no.	Best combination	Cross-validation consistency	Testing balanced accuracy	*p-values* ^*^
SNP- SNP interactions ^a^				
**2**	rs1225404 rs7903146	8/10	0.524	0.256
**3**	rs1225404 rs7903146 rs12255372	7/10	0.540	0.324
4	rs1225404 rs7903146 rs12255372 rs11196205	6/10	0.496	0.624
Gene- abdominal obesity interactions ^b^				
2	rs1225404 abdominal obesity	10/10	0.632	0.010
**3**	rs1225404 rs7903146 abdominal obesity	9/10	0.518	0.182
4	rs1225404 rs7903146 rs12255372 abdominal obesity	8/10	0.496	0.532
5	rs1225404 rs7903146 rs12255372 rs11196205 abdominal obesity	7/10	0.515	0.425

^a^Adjusted for gender, age, age at menarche, age at menopause, number of children, WC

^b^Adjusted for gender, age, age at menarche, age at menopause, number of children

**Fig. 1:** Stratified analysis for rs1225404- abdominal obesity interaction on BC risk using logistic regression

The D′ values among four *TCF7L2* gene SNPs were calculated using pairwise LD method. The results showed that value calculated for rs1225404 and rs7903146 was 0.854. Therefore, analysis for rs1225404 and rs7903146 was performed with in silico haplotype analysis by SHEsis software. As a result, the frequency of rs1225404-C and rs7903146-T haplotype was the highest in both groups (47.26% for BC patients, 54.02% for healthy controls). Also, our results demonstrated that rs1225404-T and rs7903146-C haplotype were associated with higher BC risk (Table 5).

**Table 5:** Haplotype analysis on relationship between *TCF7L2* gene and BC risk

Haplotypes (rs1225404- rs7903146)		Frequencies		OR (95%CI)	*P*-values^*^
		BC patients	Controls		
T	C	0.4726	0.5402	1.00	–
C	C	0.2243	0.2112	1.16 (0.72–1.63)	0.602
T	T	0.2019	0.1963	1.37 (0.80–1.78)	0.428
C	T	0.1012	0.0523	1.5 (1.09–2.03)	0.002

*Adjusted for gender, age, age at menarche, age at menopause, number of children, WC

## Discussion

In this study, we evaluated the effect of *TCF7L2* SNPs on BC risk. Results indicated that the BC risk of rs1225404 polymorphism C allele carriers was obviously higher than that of TT genotype carriers. Additionally, we also found that participants with rs7903146- T allele had higher BC risk than those with CC genotype. Nevertheless, after covariates adjustment, we did not discover any significant correlation among rs12255372 and rs11196205 and BC susceptibility. There was high linkage disequilibrium between rs7903146 polymorphism and rs12255372 and microsatellite DG10S478 [18]. Previous researchers have indicated that the *TCF7L2* rs7903146 polymorphism probably increase the risk of breast cancer [15, 16, 19], colorectal cancer and lung cancer [20]. SNPs of *TCF7L2* gene are considered as a risk factors for BC, and a study have shown that rs7903146 (C/T) polymorphism is associated with BC risk in Hispanic patients [15]. Another research showed a significant correlation between rs7003146 (G/T) polymorphism and reduction of BC risk in Chinese Han population [20], and rs1225404 (GA/AA genotype) was a probable anti-breast cancer factor in Hispanic population [15]. Till now, limited study focused on correlation between *TCF7L2* gene SNPs and BC risk, while just one study [21] was performed in Chinese population. Rs7903146 is located at *TCF7L2* intron region and is associated with an increased risk of BC. Variation of rs12255372 (G/T) polymorphism increases susceptibility of German familial BC [14]. Nevertheless, other studies found no correlation between rs12255372 and BC in US patients [16, 17]. And our result showed that rs12255372 minor allele was not related with BC risk. BC susceptibility was influenced by many risk factors, including genetic factors, environmental factors, and gene-environment interactions. As we all known that obesity was a risk factor for BC risk [22], Breast tissue density was higher in premenopausal women with abdominal obesity [23], and the risk of triple negative BC was increased [24, 25]. In this study, the mean WC value of BC patient group was higher than that of control group. Therefore, we also conducted *TCF7L2* gene-environment interaction between *TCF7L2* gene and abdominal obesity (defined by WC). we found a possible gene–environment interaction between rs1225404 and abdominal obesity. Compared with participants with normal WC and rs1225404- TT genotype, abdominal obese subjects with rs1225404- TC or CC genotype had the highest BC risk. Previous research showed association between others gene-obesity interaction and BC risk [26, 27], such as mutation of leptin receptor (LEP rs7799039 AA or LEPRrs1137100 GG) [26]. Long non-coding RNA and Muskelin 1 gene combined mutations was associated with high BMI and increased BC risk. As far as we know, this study was the first research to evaluate the effect of *TCF7L2* gene-abdominal obesity interaction on BC risk in Chinese population. The exact mechanism for *TCF7L2* rs1225404 gene- abdominal obesity interaction is still unclear, but we believe that *TCF7L2-* rs1225404 gene and abdominal obesity are related to BC susceptibility or BC related risk factors, the common biological mechanism is the basis of gene abdominal obesity interaction.

This research has some limitations. Firstly, the number of SNPs selected in *TCF7L2* gene is limited, and more SNPs should be selected in future research. Secondly, future research should add more environmental factors to gene-environment interaction model such as obesity, diet, life-style and activity factors. Thirdly, because of the limited sample size, we could not group the BC cases into different subtypes, and to investigate the association between SNPs and susceptibility to BC, future studies were needed to investigate the impact of more SNPs of *TCF7L2* gene on different BC subtypes. Lastly, future studies could investigate whether genotype distribution of SNP depend from clinical demographic features of studied patients.

In summary, our research shows that rs1225404 C allele and rs7903146 T allele, interaction between rs1225404 and abdominal obesity, rs1225404-T and rs7903146-C haplotypes are all related to increased risk of BC.

## Data Availability

The datasets generated and/or analyzed during the current study are available from the corresponding author on reasonable request.

## Abbreviations

OR: Odds ratios
CI: Confidence interval
TF7L2: Factor 7-like 2 gene
BC: Breast cancer
GMDR: Generalized multifactor dimensionality reduction
T2DM: Type 2 diabetes mellitus
DN: Diabetic nephropathy
SNPs: Single nucleotide polymorphism
WC: Waist circumference
